The article "Compassion Fatigue Among Practicing and Future Psychiatrists: A National Perspective" was published in 2022. Journal: Cureus.

# Compassion Fatigue Among Practicing and Future Psychiatrists: A National Perspective

**DOI:** 10.7759/cureus.25417

**Published:** 2022-05-27

**Authors:** Ahmad H Almadani, Shuliweeh Alenezi, Maha S Algazlan, Ebraheem S Alrabiah

**Affiliations:** 1 Department of Psychiatry, College of Medicine, King Saud University, Riyadh, SAU

**Keywords:** professional quality of life, burnout, psychiatric trainees, psychiatrists, compassion fatigue

## Abstract

Compassion fatigue is a set of emotions and behaviors that occur as a result of assisting a person who is suffering. Compassion fatigue, burnout, and low compassion satisfaction are all hazards that professional caregivers encounter. However, in comparison to non-medical workers, psychiatrists were found to have higher levels of compassion fatigue. We conducted a cross-sectional study that targeted all psychiatrists and psychiatric trainees enlisted in Saudi Arabia at the only registering body, the Saudi Commission for Health Specialties (SCFHS). The SCFHS approved and sent an online survey consisting of a three-section questionnaire concerning sociodemographic, personal, and professional information and the Professional Quality of Life Scale (ProQOL 5). Compassion fatigue was found at an average level in 43.2% of participants, while 56.3% had a low level. An average level of burnout was found in 65.9% of participants, while 34.1% had a low level of burnout. Of all participants, 38.9% had an elevated level of compassion satisfaction. Participants who were diagnosed with psychiatric illness showed higher burnout scores (p<0.001). Divorced or separated participants had a higher compassion satisfaction score compared with single participants. A history of psychological trauma was associated with a higher compassion fatigue score (p=0.002). These findings supported the notion of trauma as a specific risk factor for compassion fatigue. They also attested to the huge burden among psychiatrists and psychiatric trainees as part of the nature of this profession. We advise developing systematic and proactive tools to screen for trauma and to support practicing and future psychiatrists, especially those at risk of compassion fatigue.

## Introduction

Compassion fatigue (CF) is the set of emotions and behaviors that result from helping or desiring to help a suffering person. It is also an occupational hazard associated with severe emotional distress in clinical work [1]. As health care professionals are normally aware of patients’ suffering or delayed recovery, their sense of compassion toward their patients may lead to CF [2]. CF is described as a cost of caring, and it leads to desensitization to patients’ suffering and ineffective care in the form of misjudgment, clinical errors, and poor treatment planning [1-3].

In addition to “compassion fatigue,” numerous terms have been used to describe states resulting from continuous exposure to highly stressful circumstances in a professional context, such as “burnout” (BO) [4] and “secondary traumatic stress” (STS) [1]. These concepts are closely related, describing the negative impact on the quality of one’s professional life [5,6]. The definitions suffer from vagueness, however, as the terms “secondary stress” and “compassion fatigue” are often interchangeable in the literature [1,7,8]. Moreover, although CF has previously been defined as a form of burnout [9], recent literature has shown that CF, BO, and STS refer to related but distinct concepts [6]. BO is the physical, emotional, and mental exhaustion that results from prolonged work-related stress [4]. CF, in contrast, is characteristic of health care professionals; it may result from a single exposure to a traumatized patient [9].

Interestingly, CF can develop suddenly, and sufferers recover faster than those suffering from burnout [1]. However, CF and BO are linked to depersonalization, a state in which one experiences feelings of being estranged, detached, or disconnected from one’s own self [10], and to suboptimal standards of patient care [9]. CF was found to be related to decreased levels of productivity, increased sick leave, and increased likelihood of leaving the profession [11-13]. Health workers with CF suffer intrusive thoughts and feelings of distress or autonomic reactivity to reminders of the traumatic experience of the patient; numbness and avoidance; and exhaustion and fatigue [1,9,14].

Several risk factors might be responsible for the development of CF: having a personal history of traumatic events, encountering patients who have experienced trauma, absence of a support system, lack of experience, lack of balance between work and personal life, and lack of self-awareness [15,16]. However, adequate social support, personal and occupational development, and self-awareness have been shown to protect against CF [1,7,9,11,15,17-20].

Professional caregivers may be at risk of developing CF, BO, and low compassion satisfaction (CS), which is defined by the sense of pleasure experienced in helping others and the extent of support obtained from colleagues [21,22]. Psychiatrists were found to have higher levels of CF than non-medical workers, including psychologists and social workers [23,24].

Several studies have explored the prevalence of CS, BO, and STS in multiple domains and the related risk and protective factors. Multiple studies suggest that CF, which consists of STS and BO [25], is highly prevalent among health workers across different settings [21,23,26-32].

At a local level, studies exploring CF have only focused on the nurse population. In a study conducted in 2018 in Mecca, Saudi Arabia, it was concluded that a moderate risk of CF and CS was present during the special work assignment during the Hajj pilgrimage season among 542 nurses from large metropolitan hospitals. A positive correlation was found between the number of working days and CF and a negative relationship between the number of working days and CS. An association was reported between the level of competence (novice to expert) and CS and levels of BO. The results also demonstrated that CF is correlated with age, gender, education, nationality, years of experience, and competency [31]. Another study in Saudi Arabia carried out among 321 nurses in critical care in four public hospitals in 2019 examined the association between demographic variables and CF (as determined by levels of BO and CS), coping strategies, and resilience. It concluded that there are correlations between the personal characteristics of critical care nurses and levels of CF, CS, and resilience to the impact of CF [32].

Psychiatrists were reported to be at high risk of developing CF [23,24]. The characteristics of people attracted to the helping professions are the same factors that put them at risk of developing vicarious trauma and job BO [30]. To date, no research has examined CF among psychiatrists or psychiatric trainees in Saudi Arabia. The objective of our study is to examine the prevalence and predictive factors of CF in psychiatrists and psychiatric trainees in Saudi Arabia with the aim of devising a future management strategy.

## Materials and methods

Sample and setting

A cross-sectional survey was conducted across Saudi Arabia from September to November 2021. The convenience sampling method included all psychiatrists and psychiatric trainees registered on the Saudi Commission for Health Specialties (SCFHS) registry (the only registering body in Saudi Arabia). In September 2021, there were 793 physicians registered under psychiatry: 438 fully certified independent psychiatrists (consultants), 355 board-certified/eligible, and 236 psychiatric trainees (206 residents and 30 fellows).

Instruments

This study used two instruments to collect the data: a self-designed questionnaire to collect sociodemographic, work-related, and personal clinical history information, and the Professional Quality of Life Scale (ProQOL 5) to assess compassion satisfaction and compassion fatigue.

The sociodemographic questionnaire

The questionnaire consisted of three-component forms to collect: (1) demographic information about age, gender, nationality, marital status, children, the region in Saudi Arabia where the participant currently works, and if residing away from their hometown; (2) personal clinical history, including chronic medical or psychiatric illnesses and personal history of trauma; (3) professional characteristics to assess work-related demographics, including duration of experience, current position, involvement in managerial work or teaching, and satisfaction with financial income.

The Professional Quality of Life Scale

The Professional Quality of Life Scale (ProQOL) Compassion Satisfaction and Fatigue Version 5 assessed CS and CF [25]. It is a 30-item self-report tool that measures the experiences of helping others and has been in use since 1995. The ProQOL assesses both the positive and negative effects of caregiving. CS represents the positive effects, and the negative effects are seen as CF. CF is subdivided into two subscales: BO and STS. Items are evaluated on a 5-point Likert scale (from 1 = never to 5 = very often). Each subscale has a total score that can be classified as low, moderate, or high. Individual ranges are shown on each subscale, and scores beyond the limits of the range may indicate a possible risk [25]. Through psychometric testing, the ProQOL has demonstrated adequate reliability and validity [33,34]. The ProQOL is one of the most popular tools to measure CF in the literature [35].

Procedure and data collection

Ethical approval for the study was obtained from the Institutional Review Board at King Saud University, College of Medicine, Riyadh, Saudi Arabia (protocol code 21/0483, July 11, 2021). A web link to the survey was sent to all the psychiatrists and psychiatric trainees in Saudi Arabia. The nature and purpose of the study, the primary investigator’s contact information, and an explanation of the confidentiality and data anonymity policy were provided. Consent to participate was obtained by clicking on the informed-consent link. After reading the informed-consent statement, the participants clicked on “Agree” to access the study’s survey. The survey took approximately five minutes to complete. An invitation to participate in the self-administered online survey was sent via email by the SCFHS to the participants’ registered emails between the months of September and November. The online survey link was also sent to participants through WhatsApp (a messaging social media application).

Analysis

Descriptive statistics are presented using mean and standard deviation for numerical variables, while numbers and percentages are used for the categorical variables. One-way ANOVA and independent samples t-test were used to compare CF, burnout, and STS levels across different participants’ groups. Multiple linear regression was used to study the variables associated with each subscale while controlling for other variables. IBM SPSS 26 for Windows software (IBM Corp., Armonk, NY, USA) [36] was used for the analysis, and a p-value < 0.05 was considered statistically significant.

## Results

Sample characteristics and response rate

The response rate was reported to be 28.9% of the targeted sample. Of the 328 participants who filled in the survey, 99 surveys were excluded because of incomplete data, which would have affected the validity and representativeness of the sample if included. A total of 229 participants were included in this study. 63.8% of the participants were male in the whole sample, and 36.2% were females. Of the participants, 58.1% had children, while 41.9% did not have children. 74.7% of the participants were Saudi, while 25.3% were non-Saudis. Other sociodemographic characteristics are displayed in Table 1.

**Table 1:** Characteristics of participants (N = 229).

		N	%
Age	Younger than 30	70	30.6
	30–40	86	37.6
	41–50	45	19.7
	Older than 50	28	12.2
Gender	Male	146	63.8
	Female	83	36.2
Nationality	Saudi	171	74.7
	Non-Saudi	58	25.3
Marital status	Single	73	31.9
	Married	144	62.9
	Divorced or separated	12	5.2
Have Children	No	96	41.9
	Yes	133	58.1
Region where currently work/train	Central region	97	42.4
	Western region	52	22.7
	Eastern region	34	14.8
	Northern region	13	5.7
	Southern region	33	14.4
Residing away from hometown	No	127	55.5
	Yes	102	44.5
Has chronic medical illness	No	178	77.7
	Yes	51	22.3
Has psychiatric illness	No	188	82.1
	Yes	41	17.9
History of psychological trauma	No	170	74.2
	Yes	59	25.8
Position	R1-R2 (junior level of training)	54	23.6
	R3-R4 (senior level of training)	40	17.5
	Board-certified/eligible	60	26.2
	Consultants	75	32.8
Duration of experience	Less than 3 months	16	7.0
	3 months to 5 years	94	41.0
	6 years to 10 years	33	14.4
	11 years to 20 years	59	25.8
	More than 20 years	27	11.8
Involved in managerial/administrative work	No	130	56.8
	Yes	99	43.2
Involved in teaching	No	122	53.3
	Yes	107	46.7
Satisfied with financial income	No	65	28.4
	Yes	164	71.6

Reliability of measures

Cronbach’s alpha was used to test the reliability of each subscale (CF, BO, and STS). All subscales had acceptable levels of Cronbach’s alpha (Table 2).

**Table 2:** Reliability and summary of each sub-scale.

	No of Items	Mean	SD	Cronbach’s Alpha
Compassion Satisfaction	10	39.06	5.72	0.87
Burnout	10	23.41	4.76	0.66
Secondary Traumatic Stress	10	22.09	6.02	0.83

Levels of compassion satisfaction, burnout, and secondary traumatic stress

Compassion satisfaction showed high levels in 38.9% of participants; however, 59.8% had an average level and only 1.3% had a low level. None of the participants reported a high level of burnout, while 65.9% had an average level of burnout and 34.1% had a low level of burnout. Only one participant had a high level of secondary traumatic stress, while 43.2% had an average level of secondary traumatic stress and 56.3% had a low level (Table 3).

**Table 3:** Prevalence of different levels of Compassion Satisfaction, Burnout, and Secondary Traumatic Stress.

		N	%
Compassion Satisfaction	Low (22 or less)	3	1.3
	Average (Between 23 and 41)	137	59.8
	High (42 or more)	89	38.9
Burnout	Low (22 or less)	78	34.1
	Average (Between 23 and 41)	151	65.9
	High (42 or more)	0	0.0
Secondary Traumatic Stress	Low (22 or less)	129	56.3
	Average (Between 23 and 41)	99	43.2
	High (42 or more)	1	0.4

Factors associated with compassion satisfaction

To understand the relationship and the association between the different factors and the compassion satisfaction, we used independent samples t-test or one-way ANOVA, and post hoc testing was done using the Bonferroni adjustment (Table 4). The factors that showed a statistically significant association were marital status and having a history of psychiatric illness. Those who were divorced or separated had a higher compassion satisfaction score than those who were single. Not surprisingly, participants diagnosed with psychiatric illness showed a lower compassion satisfaction score than those who were not. Multiple linear regression was used to assess those variables further (Table 5). Those who were divorced or separated showed a higher compassion satisfaction score compared to those who were single by an average of 6.27 (95% CI: 2.31, 10.23), p-value = 0.002. Additionally, those diagnosed with psychiatric illnesses showed a lower compassion satisfaction score than those not diagnosed with psychiatric illnesses by an average of −3.79 (95% CI: −6.09, -1.50), p-value = 0.001.

**Table 4:** Factors associated with compassion satisfaction.

		N	Mean	SD	p-Value
Age	Younger than 30	70	38.73	5.69	0.199
	30–40	86	38.56	5.96	
	41–50	45	39.24	4.93	
	Older than 50	28	41.14	6.02	
Gender	Male	146	39.23	5.51	0.564
	Female	83	38.77	6.10	
Nationality	Saudi	171	38.98	5.86	0.702
	Non-Saudi	58	39.31	5.33	
Marital status	Single	73	37.66	6.23	0.012
	Married	144	39.47	5.40	
	Divorced or separated	12	42.75	3.84	
Have Children	No	96	38.40	5.99	0.135
	Yes	133	39.54	5.49	
Region where you currently work or train	Central region	97	38.86	5.29	0.813
	Western region	52	39.15	6.13	
	Eastern region	34	38.76	7.16	
	Northern region	13	38.31	4.48	
	Southern region	33	40.12	5.21	
Residing away from home town	No	127	38.51	5.67	0.105
	Yes	102	39.75	5.74	
Diagnosed with chronic medical illnesses	No	178	38.93	5.57	0.508
	Yes	51	39.53	6.24	
Diagnosed with psychiatric illnesses	No	188	39.60	5.14	0.018
	Yes	41	36.61	7.45	
History of psychological trauma	No	170	39.01	5.40	0.823
	Yes	59	39.22	6.60	
Position	R1-R2 (junior level of training)	54	38.48	5.94	0.350
	R3-R4 (senior level of training)	40	38.63	6.46	
	Board-certified/eligible	60	38.65	4.96	
	Consultants	75	40.04	5.70	
Duration of experience	Less than 3 months	16	39.44	6.429	0.233
	3 months to 5 years	94	38.27	6.119	
	6 years to 10 years	33	39.73	4.404	
	11 years to 20 years	59	38.95	5.158	
	More than 20 years	27	41.04	6.236	
Involved in managerial/administrative work	No	130	39.06	5.81	0.999
	Yes	99	39.06	5.63	
Involved in teaching	No	122	38.79	5.91	0.440
	Yes	107	39.37	5.51	
Satisfied with financial income	No	65	38.26	4.56	0.133
	Yes	164	39.38	6.10	

**Table 5:** Multiple linear regression for the factors associated with Compassion Satisfaction. * Ref = Reference category.

	Compassion Satisfaction			
	Coefficient	p-Value	[95% Confidence Interval]	
Age				
Younger than 30	Ref *			
30–40	−1.57	0.216	−4.07	0.93
41–50	−1.34	0.456	−4.88	2.20
Older than 50	−0.43	0.865	−5.45	4.59
Gender				
Male	Ref *			
Female	−0.26	0.768	−1.97	1.46
Nationality				
Saudi	Ref *			
Non-Saudi	−1.80	0.122	−4.09	0.49
Marital status				
Single	Ref *			
Married	1.82	0.254	−1.32	4.96
Divorced or separated	6.27	0.002	2.31	10.23
Have Children				
No	Ref *			
Yes	−0.93	0.52	−3.79	1.92
Region in Saudi				
Central	Ref*			
Western region	0.37	0.709	−1.60	2.35
Eastern region	−0.18	0.878	−2.53	2.16
Northern region	−1.09	0.522	−4.45	2.27
Southern region	1.66	0.175	−0.74	4.07
Residing away from hometown				
No	Ref *			
Yes	1.79	0.034	0.13	3.44
Diagnosed with chronic medical illnesses				
No	Ref *			
Yes	0.23	0.826	−1.81	2.27
Diagnosed with psychiatric illnesses				
No	Ref *			
Yes	−3.79	0.001	−6.09	−1.50
Personal history of psychological trauma				
No	Ref *			
Yes	1.47	0.164	−0.60	3.54
Position	Ref *			
R1-R2 (junior level of training)				
R3-R4 (senior level of training)	0.26	0.849	−2.43	2.95
(Board-certified awaiting independent license)	0.78	0.629	−2.39	3.95
Consultants (independent license)	1.53	0.437	−2.34	5.40
Duration of experience				
Less than 3 months	Ref *			
3 months to 5 years	−1.05	0.532	−4.38	2.27
6 years to 10 years	1.19	0.586	−3.12	5.50
11 years to 20 years	−0.09	0.97	−4.64	4.47
More than 20 years	0.74	0.81	−5.33	6.81
Involved in managerial (or administrative) work				
No	Ref *			
Yes	−0.56	0.561	−2.44	1.33
Involved in teaching				
No	Ref *			
Yes	−0.32	0.75	−2.32	1.67
Satisfied with financial income				
No	Ref *			
Yes	1.10	0.214	−0.64	2.85

Factors associated with burnout

Using the same factors and statistical methods for CS, we examined the association between those factors and burnout (Table 6). Factors that showed statistically significant association were age, gender, satisfaction with financial income, and having a history of psychiatric illness (for the same findings in a multiple linear regression model, see Table 7). Those in the age group 30-40 had higher burnout scores compared to those older than 50. Interestingly, females had a higher burnout score compared to males. Furthermore, participants diagnosed with psychiatric illness showed higher burnout scores than those who were not. Those who were not satisfied with their financial income had higher burnout scores compared to those who were satisfied.

**Table 6:** Factors associated with burnout.

		N	Mean	SD	p-Value
Age	Younger than 30	70	23.59	4.29	0.021
	30–40	86	24.06	4.73	
	41–50	45	23.36	4.69	
	Older than 50	28	21.04	5.54	
Gender	Male	146	22.86	4.70	0.020
	Female	83	24.37	4.73	
Nationality	Saudi	171	23.51	4.66	0.576
	Non-Saudi	58	23.10	5.07	
Marital status	Single	73	24.12	4.47	0.287
	Married	144	23.04	4.88	
	Divorced or separated	12	23.42	4.85	
Have Children	No	96	23.98	4.32	0.122
	Yes	133	22.99	5.03	
Region in Saudi Arabia where you currently work or train	Central region	97	23.26	4.36	0.959
	Western region	52	23.19	4.92	
	Eastern region	34	23.82	5.10	
	Northern region	13	23.38	4.48	
	Southern region	33	23.76	5.56	
Residing away from hometown	No	127	23.35	4.93	0.833
	Yes	102	23.48	4.55	
Diagnosed with chronic medical illnesses	No	178	23.42	4.47	0.937
	Yes	51	23.35	5.70	
Diagnosed with psychiatric illnesses	No	188	22.88	4.55	<0.001
	Yes	41	25.80	5.03	
History of psychological trauma	No	170	23.21	4.54	0.295
	Yes	59	23.97	5.33	
Position	R1-R2 (junior level of training)	54.00	23.48	4.10	0.200
	R3-R4 (senior level of training)	40.00	24.58	5.01	
	Board-certified/eligible	60.00	23.57	4.39	
	Consultants	75.00	22.60	5.26	
Duration of experience	Less than 3 months	16	23.00	4.274	0.062
	3 months to 5 years	94	23.96	4.529	
	6 years to 10 years	33	23.06	4.847	
	11 years to 20 years	59	23.92	4.481	
	More than 20 years	27	21.04	5.754	
Involved in administrative work	No	130	23.38	4.58	0.916
	Yes	99	23.44	5.01	
Involved in teaching	No	122	23.67	4.24	0.374
	Yes	107	23.10	5.29	
Satisfied with financial income	No	65	24.54	4.50	0.023
	Yes	164	22.96	4.80	

**Table 7:** Multiple linear regression for the factors associated with Burnout. * Ref = Reference category.

	Burnout			
	Coefficient	p-Value	[95% Confidence Interval]	
Age				
Younger than 30	Ref *			
30–40	0.6	0.575	−1.51	2.7
41–50	−0.16	0.917	−3.14	2.82
Older than 50	−0.71	0.741	−4.93	3.52
Gender				
Male	Ref *			
Female	1.22	0.096	−0.22	2.66
Nationality				
Saudi	Ref *			
Non-Saudi	1	0.306	−0.92	2.93
Marital status				
Single	Ref *			
Married	−0.04	0.975	−2.68	2.6
Divorced or separated	−1.64	0.332	−4.97	1.69
Have Children				
No	Ref *			
Yes	−0.29	0.811	−2.7	2.11
Region in Saudi				
Central	Ref *			
Western region	−0.22	0.798	−1.88	1.45
Eastern region	0.45	0.653	−1.52	2.42
Northern region	0.16	0.912	−2.67	2.99
Southern region	0.31	0.766	−1.72	2.33
Residing away from hometown				
No	Ref *			
Yes	0.08	0.907	−1.31	1.48
Diagnosed with chronic medical illnesses				
No	Ref *			
Yes	0.6	0.489	−1.11	2.32
Diagnosed with psychiatric illnesses				
No	Ref *			
Yes	2.64	0.008	0.71	4.57
Personal history of psychological trauma				
No	Ref *			
Yes	−0.45	0.611	−2.2	1.29
Position	Ref *			
R1-R2 (junior level of training)				
R3-R4 (senior level of training)	0.82	0.474	−1.44	3.09
(Board-certified awaiting independent license)	−0.43	0.753	−3.09	2.24
Consultants (independent license)	−0.61	0.713	−3.86	2.65
Duration of experience				
Less than 3 months	Ref *			
3 months to 5 years	1.33	0.349	−1.47	4.13
6 years to 10 years	0.75	0.683	−2.88	4.38
11 years to 20 years	1.92	0.325	−1.91	5.75
More than 20 years	−0.13	0.959	−5.24	4.98
Involved in managerial (or administrative) work				
No	Ref *			
Yes	0.79	0.324	−0.79	2.38
Involved in teaching				
No	Ref *			
Yes	−0.48	0.574	−2.16	1.2
Satisfied with financial income				
No	Ref *			
Yes	−1.18	0.116	−2.65	0.29

Factors associated with secondary traumatic stress

We also assessed the factors associated with secondary traumatic stress (Table 8). Nationality, a history of psychiatric illness, and a personal history of psychological trauma all exhibited statistically significant associations. In comparison to Saudi participants, non-Saudi participants had a higher secondary traumatic stress score. In comparison to those who were not diagnosed with a psychiatric disorder, those who were showed a higher secondary traumatic stress score. Participants who had experienced psychological trauma in the past scored higher on secondary traumatic stress than those who had not (Table 9).

**Table 8:** Factors associated with Secondary Traumatic Stress.

Age	Younger than 30
	30–40
	41–50
	Older than 50
Gender	Male
	Female
Nationality	Saudi
	Non-Saudi
Marital status	Single
	Married
	Divorced or separated
Have Children	No
	Yes
Region in Saudi Arabia where you currently work or train	Central region
	Western region
	Eastern region
	Northern region
	Southern region
Residing away from hometown	No
	Yes
Diagnosed with chronic medical illnesses	No
	Yes
Diagnosed with psychiatric illnesses	No
	yes
History of psychological trauma	No
	Yes
Position	R1-R2 (junior level of training)
	R3-R4 (senior level of training)
	Board-certified/eligible
	Consultants
Duration of experience	Less than 3 months
	3 months to 5 years
	6 years to 10 years
	11 years to 20 years
	More than 20 years
Involved in administrative work	No
	Yes
Involved in teaching	No
	Yes
Satisfied with financial income	No
	Yes

**Table 9:** Multiple linear regression for the factors associated with Secondary Traumatic Stress. * Ref = Reference category.

	Secondary Traumatic Stress (Compassion Fatigue)			
	Coefficient	p-Value	[95% Confidence Interval]	
Age				
Younger than 30	Ref *			
30–40	−1.21	0.372	−3.87	1.45
41–50	−1.12	0.559	−4.89	2.65
Older than 50	−2.28	0.401	−7.63	3.07
Gender				
Male	Ref *			
Female	1.29	0.164	−0.53	3.12
Nationality				
Saudi	Ref *			
Non-Saudi	2.51	0.044	0.07	4.95
Marital status				
Single	Ref *			
Married	1.72	0.312	−1.62	5.06
Divorced or separated	2.02	0.345	−2.19	6.24
Have Children				
No	Ref *			
Yes	−0.86	0.578	−3.9	2.18
Region in Saudi				
Central	Ref *			
Western region	0.32	0.765	−1.78	2.42
Eastern region	0.76	0.549	−1.74	3.25
Northern region	0.88	0.628	−2.7	4.46
Southern region	1.87	0.152	−0.69	4.44
Residing away from hometown				
No	Ref *			
Yes	−0.27	0.76	−2.04	1.49
Diagnosed with chronic medical illnesses				
No	Ref *			
Yes	0.87	0.433	−1.31	3.04
Diagnosed with psychiatric illnesses				
No	Ref *			
Yes	1.31	0.291	−1.13	3.75
Personal history of psychological trauma				
No	Ref *			
Yes	2.34	0.038	0.13	4.54
Position				
R1-R2 (junior level of training)	Ref*			
R3-R4 (senior level of training)	1.22	0.402	−1.64	4.08
(Board-certified awaiting independent license)	−0.54	0.751	−3.92	2.83
Consultants (independent license)	−0.78	0.708	−4.9	3.33
Duration of experience				
Less than 3 months	Ref *			
3 months to 5 years	−0.13	0.943	−3.67	3.41
6 years to 10 years	2.33	0.317	−2.26	6.92
11 years to 20 years	2.62	0.288	−2.23	7.46
More than 20 years	1.73	0.598	−4.73	8.2
Involved in managerial (or administrative) work				
No	Ref *			
Yes	0.44	0.668	−1.57	2.44
Involved in teaching				
No	Ref *			
Yes	−1.2	0.268	−3.32	0.93
Satisfied with financial income				
No	Ref *			
Yes	−0.44	0.643	−2.3	1.42

## Discussion

This is the first study to report on CF and associated factors in psychiatrists and future psychiatrists in Saudi Arabia. The main goal of CF research is to maintain healthier care providers who can apply the principles of resiliency and quickly recover to high-functioning behaviors, both at work and outside of work, after being exposed to a patient’s or client’s traumatic event. Although percentages of CF were not high in this report, which was very reassuring, our findings still supported the notion of secondary traumatic stress being closely associated with high levels of burnout [37]. In our study, 99 (43.2%) of the participants experienced an average level of CF, while 129 (56.3%) had a low level of CF. CF in our study was found to be much lower than levels of CF found in other studies [21,23,26,27]. However, our finding was consistent with a study on cardiac physicians in a culturally related country, Pakistan [38].

We found that female psychiatrists and psychiatric trainees were more prone to score higher on the burnout domain scores than males, which agreed with a study conducted among family practitioners in Israel [21]. The reverse was found among nurses, where burnout rates were lower in females than in males [39], which was explained by culturally dictated gender roles [32]. In addition, younger physicians showed higher burnout scores than those older than 50 years. This finding was similar to studies done in Pakistan [38] and the UK [23]. It can be attributed to less professional experience, subsequent increased work-related stress [26], and lack of experience in coping with work-related stress [38]. Another alternative explanation may be the huge workload in the earlier years of the profession. Moreover, satisfaction with financial income was significantly associated with lower burnout scores. Regarding having children, this could not be identified as a protective factor against BO in our study, which disagreed with a study by Haik among burn-unit clinicians that found that having children decreases the risk of developing BO and CF and justified children as a source of emotional support and distraction from work-related stress [26].

Compassion satisfaction was significantly correlated with marital status, as divorced or separated participants showed a higher compassion satisfaction than those who were single, which was inconsistent with the results of a study in Israel suggesting that divorced participants are at greater risk of developing CF than single participants [26]. This finding appeared surprising. However, it may be seen as compensation for a perceived failure in one aspect of life. Further research is needed to explore it. Interestingly, doctors who reside away from home scored higher on the compassion satisfaction score, which has never been assessed in relation to compassion satisfaction in other studies, to our knowledge. More research is needed to ascertain the impact of residing away from home on compassion satisfaction and compassion fatigue.

Consistent with the study in the UK [23] and Dallas, US [28], a personal history of psychological trauma was found to be a significant risk factor for the development of CF. Research has suggested that therapists with a previous history of trauma are vulnerable to the trauma stories of others [40]. No correlation between personal trauma and BO was found in our study, unlike the finding in a study in Israel [21]. In contrast to a study in the US [29], we found no association between the female gender and CF.

Notably, in the three domains of CF, BO, and CS, diagnosis of psychiatric illness was significant and were found to have higher levels of BO and CF and lower levels of CS. Surprisingly, the position of psychiatrist and psychiatric trainee (including his/her level in residency) and duration of experience showed no significant association with any of the domains mentioned above. This contradicted the findings of a study among nurses that showed a negative relationship between years of experience and CF [31]. Furthermore, holding managerial positions and being teaching residents had no impact on CS, which was inconsistent with the study in Israel [21] that linked both of them with higher CS.

Limitations and future directions

Despite representing a fair response rate, our sample population was limited as it focused only on psychiatrists and psychiatric trainees. The cross-sectional nature of our study limited our ability to assess the prevalence of compassion fatigue longitudinally. A large-scale study of compassion fatigue among other mental health professionals such as psychologists and social workers could further understand the phenomena of compassion fatigue. Moreover, a qualitative approach could help explore psychiatrists' and psychiatric trainees’ perceptions of compassion fatigue and study protective measures to be utilized by doctors and hospitals if consistent reports of low CF were present.

## Conclusions

Our findings supported the notion of trauma as a specific risk factor for compassion fatigue. We also found that burnout was more common in female psychiatrists and psychiatric trainees than in males. Psychiatrists who were divorced or separated had more compassion satisfaction than those who were single. Additionally, a personal history of psychological trauma was a considerable risk factor for compassion fatigue development. We suggest the Saudi Medical Association develop systematic and proactive tools to screen for trauma and support practicing and future psychiatrists at risk of compassion fatigue.
